# Identification and Functional Analysis of the Sex-Determiner *Transformer-2* Homologue in the Freshwater Pearl Mussel, *Hyriopsis cumingii*

**DOI:** 10.3389/fphys.2021.704548

**Published:** 2021-07-08

**Authors:** Yayu Wang, Xiaoqiang Wang, Jingyuan Ge, Guiling Wang, Jiale Li

**Affiliations:** ^1^Key Laboratory of Freshwater Aquatic Genetic Resources, Ministry of Agriculture and Rural Affairs, Shanghai Ocean University, Shanghai, China; ^2^National Demonstration Center for Experimental Fisheries Science Education, Shanghai, China; ^3^Shanghai Engineering Research Center of Aquaculture, Shanghai, China

**Keywords:** *Hyriopsis cumingii*, *transformer-2*, gonadal development, sex determination, *in situ* hybridization, RNA interference

## Abstract

*Transformer-2 (Tra-2)* is an upstream regulatory element of the sex regulation mechanism in insects and plays a critical role in sex formation. To understand the role of *tra-2* in *Hyriopsis cumingii*, the full-length *Hctra-2* (1867 bp) was obtained from the gonads, and sequence alignment with other species showed that HCTRA-2 protein had a highly conserved RRM domain. Phylogenetic analysis showed that the HCTRA-2 protein was a close relative to of the mollusks TRA-2 protein. The qRT-PCR of tissue-specific expression pattern showed that the *Hctra-2* was abundant in gonads, and the expression in testes was higher than that in ovaries (*p* < 0.01). It suggests that *Hctra-2* may play a potential regulatory role in gonadal development of *H. cumingii*. In the early gonadal development, the *Hctra-2* expression was the highest on the third day after fertilization and increased slightly from 4 months to 5 months, which may be related to the embryonic sex determination and early gonadal development. *In situ* hybridization showed that *Hctra-2* mRNA signals were present in both male and female gonads. After silencing *Hctra-2* by RNAi, the expression levels of *Hcfem-1b* and *Hcdmrt* were changed. It is speculated that there may be a certain relationship between them, which plays an important role in the sex regulation of *H. cumingii*. Our research will help to deepen our understanding of the shellfish sex determination mechanisms.

## Introduction

*Hyriopsis cumingii* is a pearl-cultured species unique to China. The pearl cultivated by it has smooth and delicate nacre quality and bright color, which is the best one among freshwater mussels (Wang et al., 2007). Interestingly, male and female mussels showed different traits in the culture, and the quality of pearl produced by males was better than that of females (Zhao et al., 2013). Therefore, it is of great significance to raise the pearl yield and quality by using sex control technology. However, the research on the regulation mechanism of *H. cumingii* sex determination is limited, which hinders the development of sex control breeding technology.

In shellfish, there are androgyny, hermaphroditism, or sex reversal in their sex (Yue et al., 2020). This complex and changeable sex type provides us with a lot of rich research resources and brings some challenges to the study of sex. In recent years, the rapid development of sequencing technology has brought new hope to shellfish sex research. Some genes related to sex determination and differentiation have also been identified in shellfish, such as *foxl2*, *tra*, *dmrt*, *fem-1*, *soxe*, *soxh*, and *wnt4* (Naimi et al., 2009; Shi et al., 2015, 2018; Li et al., 2016; Galindo-Torres et al., 2018). Among these genes, the *tra* was an upstream component of the sex-regulatory mechanism in many species, playing a crucial role in the regulation of sex formation mechanisms. In *Caenorhabditis elegans*, *tra-1* and *tra-2* promote female fates (Wang and Kimble, 2001). The regulatory pathway of sex determination is mainly composed of *her-1*, *tra-2*, *fem-1*, *fem-2*, *fem-3*, and *tra-1*. The specific regulatory mechanism is as follows: the ratio of sex chromosome and autosome is the primary signal of sex regulation (Farboud et al., 2013). The signal acts on *her-1*, which is differentially expressed between two genders. In male XO individuals, *her-1* expression is very high, which inhibits the transmembrane receptor protein of TRA-2. Then, the complex formed by the proteins of FEM-1, FEM-2, FEM-3, and CUL-2 binds with the specific site of *tra-1*, which makes the individual develop into male. In XX hermaphrodite, *her-1* expression is very low or even not expressed, so the TRA-2 protein is active. The combination of TRA-2 and the complex containing FEM-1, FEM-2, and FEM-3 proteins makes the expression of TRA-1 protein, and the organism develops toward hermaphroditism (Kuwabara, 2007; Starostina et al., 2007; Mapes et al., 2010). In Drosophila, the regulation of sex is as follows: X: A > *sex lethal* (*sxl*) > *tra*/*tra-2* > *doublesex* (*dsx*), and *fruitless* (*fru*) (Suzuki, 2010). Sex determination is determined by the ratio of X chromosome number to autosomal number. In females, the presence of two X chromosomes activated the expression of *sxl*. Subsequently, *sxl* regulates the splicing of *tra* pre-mRNA transcripts to produce RNA encoding full-length and functional TRA proteins (Sosnowski et al., 1989). Together with *tra-2*, *tra* promotes female-specific splicing of *dsx* and prevents *fru* synthesis (Camara et al., 2019). In drones, the *sxl* is inactivated, resulting in the lack of active TRA proteins. Therefore, *dsx* and *fru* precursor mRNA default to male-specific splicing, and ontogeny is male (Grmai et al., 2018).

In aquatic species, there are few studies on *tra-2*, and its action on sex is not clear. In *Macrobrachium nipponense*, *Mntra-2a* was highly expressed in both male and female gonads, and its expression was located in oocytes and spermatocytes. It may play an important role in the embryonic development and early gonadal development (Wang et al., 2019). In *Fenneropenaeus chinensis*, *Fctra-2c* may participate in female sex determination in a concentration-dependent manner (Li et al., 2012). In medaka (*Oryzias latipes*), *tra-2* transcripts (*tra-2a* and *tra-2b*) were mainly expressed in hermaphroditic germ cells before and during their sex differentiation, indicating that both *tra2a* and *tra2b* may be involved in the sex differentiation (Shiraishi et al., 2004). *Cqtra-2* may play a role in sexual differentiation in the redclaw crayfish (*Cherax quadricarinatus*), which is mainly expressed in the ovary and gradually increases with embryonic development (Cai et al., 2020).

In this study, we identified *Hctra-2* in *H. cumingii* and analyzed their expression distribution in different tissues and developmental stages of males and females. Besides, the effect of *Hctra-2* silencing *via* RNAi on the expression of *Hcfem-1b* and *Hcdmrt* was investigated. These results will be helpful to understand the sex regulation mechanism of *H. cumingii*, and provide a basis for exploring the sex of shellfish.

## Materials and Methods

### Animals and Sample Preparation

All the samples used in the study (including juveniles at different developmental stages and mature mussels) were from Zhejiang Weiming aquaculture farm. All experimental processes were approved by the Institutional Animal Care and Use Committee (IACUC) of Shanghai Ocean University, Shanghai, China.

The samples were taken back from the farm to the laboratory and placed in the water at 26 ± 2°C for 3 days. The gonads, gills, liver, kidney, mantle, foot, and adductor tissues of adult mussels were collected. Embryonic samples were scraped from the gills of *H. cumingii* at 1 day, 3 days, 5 days, 7 days, 9 days, and 10 days after fertilization. In the juvenile, samples were taken periodically according to different ages. All samples were immediately frozen in liquid nitrogen and stored at - 80°C for RNA extraction.

### Full-Length Cloning of *Hctra-2*

*Hctra-2* was derived from the transcriptome library. First, we verified the correctness of partial *Hctra-2* sequence. Total RNA was extracted from frozen tissues with RNA prep pure tissue Kit (Tiangen, China). The cDNA was synthesized according to the manufacturer’s protocol of the PrimeScript RT reagent Kit with gDNA Eraser kit (TaKaRa, Japan). Using Tra-F and Tra-R (Table 1) as primers, the sequence of *Hctra-2* was amplified by PCR under the following conditions: 94°C for 3 min, followed by 35 cycles of 95°C for 30 s denaturation, 55°C for 30 s of annealing, and 72°C for 2 min extension. After PCR, the amplified targeted-DNA was subcloned into the pMD19 vector (TaKaRa, Japan) for sequence confirmation. The full-length cDNA sequence of *Hctra-2* was amplified by the SMARTer RACE 5'/3' Kit (Clontech, United States). The primers used for race amplification were T2-3' and T2-5', and the sequences are shown in Table 1. The reaction products obtained from the RACE kit instructions were purified by 1% agarose gel electrophoresis and connected to the carrier pMD19 vector and then transformed into *Escherichia coli* DH5α competent cells. Finally, the positive clones were screened for sequencing. Splicing 3' and 5' sequences to obtain the full-length sequence of *Hctra-2*.

**Table 1:** Primers for the present study.

Name	Sequences (5'-3')	Application
Tra-F	CTTCCAGGACACCCTCAAGGTCAAG	Verification
Tra-R	GGAGCGTTTCCTACTGAATCC	sequence
T2-3'	GATAGATGGTAGAAGAATCAGGGT	3' RACE
T2-5'	CGTGAATGTTTGTGGTGTTCTCTGCTTT	5' RACE
qT2-F	TCACGAACTCCTTCCAGGAC	qRT-PCR/ISH
qT2-R	CCTGGATCTCCTCCTCCTCT	qRT-PCR/ISH
EFl-αF	GGAACTTCCCAGGCAGACTGTGC	qRT-PCR
EFl-αR	TCAAAACGGGCCGCAGAGAAT	qRT-PCR
qfem-1b-F	TCACTTTGGAGTCGTCAGGC	qRT-PCR
qfem-1b-R	CAGGTACCGCACAATGTCGT	qRT-PCR
qdmrt-F	CCGAAACCATGGCGTTGTAT	qRT-PCR
qdmrt-R	CTTGAGCCTGTTGCCTTCTC	qRT-PCR
IT2-F	TAATACGACTCACTATAGGGTCACGAACTCCTTCCAGGAC	ISH
IT2-R	TAATACGACTCACTATAGGGCCTGGATCTCCTCCTCCTCT	ISH
T2-RNAi-F1	GTCCCGAAGCCCCTATT	RNAi
T2-RNAi-R1	TAATACGACTCACTATAGGGCCACCCTGATTCTTCTACCA	RNAi
T2-RNAi-F2	TAATACGACTCACTATAGGGGTCCCGAAGCCCCTATT	RNAi
T2-RNAi-R2	CCACCCTGATTCTTCTACCA	RNAi
GFP-RNAi-F1	AAGGGCGAGGAGCTGTTCACCG	RNAi
GFP-RNAi-R1	TAATACGACTCACTATAGGGCAGCAGGACCATGTGATCGCGC	RNAi
GFP-RNAi-F2	TAATACGACTCACTATAGGGAAGGGCGAGGAGCTGTTCACCG	RNAi
GFP-RNAi-R2	CAGCAGGACCATGTGATCGCGC	RNAi

### Bioinformatics Analysis of *Hctra-2*

The open reading frame (ORF) Finder program performs^1^ open reading frame determination and amino acid sequence acquisition of *Hctra-2*. The nucleotide and amino acid sequence similarity between *Hctra-2* sequence and homologous species was analyzed by BLAST program^2^; TMHMM Server v2.0 program^3^ predicted transmembrane structure of prediction protein; SignalP 4.1^4^ predicted the presence and the location of signal peptides in prediction protein; ProtParam program^5^ predicted various physical and chemical parameters of protein; and ClustalW 1.8 and BioEdit were used for multiple comparisons of amino acid and coding nucleotide sequences. The phylogenetic tree was constructed by Neighbor-joining (NJ; Zhang and Sun, 2008) method in Mega 6.0, and the confidence values among species were calculated by Bootstrap repeated 1,000 times (Zhang and Sun, 2008).

### Expression Studies of *Hctra-2*

Quantitative real-time reverse transcription PCR was used to analyze the expression level of *Hctra-2* in different tissues and years of *H. cumingii*. The *EF-lα* was used as the internal reference. qT2-F and qT2-R were used as primers. cDNA synthesis and quantification of each mixed sample were performed using PrimeScript RT reagent Kit with gDNA Eraser kit (TaKaRa, Japan) and TB Green Premix Ex Taq II (Takara, Japan), respectively. The total qRT-PCR volume of 20 ul contained 10 ul TB Green Premix Ex Taq, 0.8 ul forward primer, 0.8 ul reverse primer, 6.8 ul ddH_2_O, and 1.6 ul cDNA. Amplification was performed using a BIO-RAD CFX96 instrument under the following conditions: pre-denaturation at 95°C for 15 min, degeneration at 95°C for 10 s, annealing at 60°C for 30 s (40 cycles), collecting signals during the extension phase, and each cycle increased 0.5°C for 5 s from 65°C to 95°C, followed collecting the fluorescence signal of the dissolution curve. The target gene and reference gene’s relative expression level was calculated using 2 ^−△△CT^ method with three replicates for each group. Use Prism 8.0 software to draw pictures. T-test calculated significant difference; *p* < 0.05 was considered statistically significant.

### *In situ* Hybridization

In the experimental group, the probe primers of *Hctra-2* were qT2-F and IT2-R (Table 1). In the control group, the probe primers were IT2-F and qT2-R (Table 1). *In vitro* transcription was performed using a T7 High Efficiency Transcription Kit (Transgen, China). DIG RNA Labeling Mix was used for probe labeling. Samples of mature gonads (male and female; 2 years old) were fixed twice in 4% paraformaldehyde, then transferred to 20% sucrose solution, sliced with a cryo slicer, and stored at −20°C. *In situ* hybridization was performed according to the Enhanced Sensitive ISH Detection Kit II (Boster, United States). Hybridization signals were observed and photographed under the microscope.

### Knockdown of *Hctra-2* by dsRNA-Mediated RNA Interference

Double-stranded RNA (dsRNA) of *Hctra-2* was prepared for the experiment of *H. cumingii* injection. The primers were dsTra-F1, dsTra-R1, dsTra-F2, and dsTra-R2 (Table 1). Firstly, the target sequence was obtained by PCR amplification, and the single-stranded RNA (ssRNA) was synthesized by T7 transcription kit *in vitro*. Then, dsRNA was synthesized according to the Ribo RNAMax-T7 *in vitro* transcription kit. The steps are as follows: mix the same amount of ssRNA into the PCR instrument and heat at 70°C for 10 min resulted in the binding of two reverse complementary ssRNAs to form dsRNA. The excess ssRNA was removed according to the procedure of Ribo RNAMax-T7, and dsRNA was dissolved in 1 × PBS. The control dsRNA was GFP sequence which had no homology with *Hctra-2*, and the primer sequence is shown in Table 1.

The experiment was divided into two groups: the experimental and the control groups, each with 10 mussels. Farm them in plastic bins. On day 1, day 6, and day 11, 100 μl (400 ng/μl) *Hctra-2* dsRNA was injected into the adductor of *H. cumingii* using a microsyringe of 1 ml, respectively. RNA was extracted from gonads, and the expression of *Hctra-2*, *Hcfem-1b*, and *Hcdmrt* after injection of *Hctra-2* dsRNA was detected by qRT-PCR. The primers for *Hcfem-1b* and *Hcdmrt* were designed based on the sequencing information of the transcriptome data of *H. cumingii*. The details are shown in Table 1.

## Results

### Molecular Identification of *Hctra-2* and Sequence Analysis

A partial sequence (about 600 bp) of *Hctra-2* cDNA was amplified by PCR using primers Tra-F and Tra-R. Based on the cDNA sequence, 5' and 3' RACE gene-specific primers (T2-3' and T2-5') were designed to amplify the 3' and 5' untranslated region sequence. After sequence splicing, the *Hctra-2* full-length cDNA 1867 bp (GenBank no. MH931228) was obtained, in which the ORF was 894 bp, the 5' untranslated region (UTR) was 92 bp, and the 3' UTR was 881 bp (Figure 1). The ORF of *Hctra-2* was predicted to encode a protein with 297 amino acids with a predicted molecular weight of 34661.2 and a theoretical isoelectric point of 11.02. The protein has no signal peptide or transmembrane structure. The 65–125 amino acid of *Hctra-2* protein is the SR1 domain, and the 128–226 amino acid is a conserved RNA recognition motif (RRM) domain, followed by the linker region (amino acid position 227–243; Figure 1).

**Figure 1:** Nucleotide and deduced amino acid sequence of *Hctra-2* gene from *Hyriopsis cumingii*. Lowercase indicated 3' and 5' UTRs; uppercases was coding region, where the upper indicated the nucleotides sequence and the lower showed the amino acids. ^*^Represented stop codon; putative polyadenylation signals (AATAAA) were underlined. The gray region was the RRM domain. The green region shows the SR1 domain. The blue region shows the linker.

### Multiple Alignment and Phylogenetic Analysis

The amino acid sequence of *Hctra-2* was analyzed by blast. The results showed that the similarity of *Hctra-2* among different species was high (65–79%), among which *Mizuhopecten yessoensis* (79.66%) was the highest. Even in humans and mice, the sequence similarity reached 69.6 and 54.7%. TRA-2 sequences of *Mytilus coruscus* (CAC5410763.1), *Crassostrea gigas* (XP_034314418.1), *M. yessoensis* (OWF38207.1), and *Pecten maximus* (XP_033761757.1) were selected from NCBI database. ClustalW in BioEdit software was used to compare the multi-sequence alignment of TRA-2. The alignment results showed that the TRA-2 of most shellfish was composed of about 300 amino acids (Figure 2), all of which contained the RRM domain, which was highly conserved and located in the same position. Similar to other species, the ribonucleoprotein 1 (RNP-1) has also been found in HCTRA-2, which is very conserved in RRM proteins (Shiraishi et al., 2004; Hu et al., 2020). Phylogenetic tree analysis showed that TRA-2 protein of *H. cumingii* clustered with *C. gigas*, *M. coruscus,* and other bivalves. Mollusks, such as *Octopus sinensis* and *Sepia pharaonis*, are classified with fish and mammals (Figure 3).

**Figure 2:** Multiple alignment of *Hctra-2* amino acid sequence from *H. cumingii* with other species. Identical amino acid residues are highlighted in black, and similar amino acids are highlighted in gray. ^*^Means that the amino acids at this site are the same in all the species compared.

**Figure 3:** NJ phylogenetic tree of amino acid sequences of *Hctra-2* gene in different species. NJ law contribution was made by MEGA6.0; the number on the node was bootstrap test confidence value repeated 1,000 times.

### Tissue-Specific Distribution of *Hctra-2* in Adult

Quantitative real-time reverse transcription PCR was performed using primers spanning the ORF of *Hctra-2*. In all tissues of female mussels, the expression of *Hctra-2* was high in gonad and liver, followed by gill and kidney, and lower in adductor, mantle, and foot. In male mussels, the expression of *Hctra-2* was higher in gonad and liver, then in adductor and gill, and lower in kidney, mantle, and foot. Compared with male and female mussels, except for kidney and foot, the expression of *Hctra-2* was significantly different (*p* < 0.05), especially in gonad, liver, adductor muscle, and mantle (*p* < 0.01; Figure 4).

**Figure 4:** Tissues expression of *Hctra-2* gene in adult male and female *H. cumingii*. Results are expressed as mean ± SD, and significance of comparison is defined as *p* < 0.05 (^*^) or *p* < 0.01 (^**^) by Student’s *t*-tests.

### Expression Pattern in Different Developmental Stages of Embryos and Juveniles

*Hctra-2* expression at different developmental stages in embryos and juveniles (from the fertilized egg up to 8 months old) was detected. The results showed that the expression of *Hctra-2* was high in the fertilized eggs, then reached the highest level on the third day, decreased rapidly on the sixth day, and remained at a low steady level until 3 months old. The *Hctra-2* expression level increased slightly at the age of 4 to 5 months old and tended to be stable at 6 months old (Figure 5).

**Figure 5:** Relative expression of *Hctra-2* gene in different developmental periods. (D: days; 0–10 days is embryonic period; M: months; 1–8 mouths is Juveniles).

### Localization of *Hctra-2* in Mature Gonads

Cell localization of *Hctra-2* in testis and ovary was detected by *in situ* hybridization. Figures 6A,D show the testes and ovaries morphology of *H. cumingii* stained with HE (hematoxylin-eosin). The male germ cells (from spermatogonia to mature sperm) and female germ cells (from oocyte to mature egg) at different developmental stages can be seen in the figure. Figures 6B,C are the control group and the experimental group of male mussels, respectively. Compared with the control group, the *Hctra-2* mRNA purple signals in the experimental group were obvious, and the signals were located on spermatogonia and spermatocytes, but no signal was found on spermatids and sperms. Figures 6E,F are the control group and the experimental group in the female gonad, respectively. Compared with the control group, the hybridized signal of *Hctra-2* mRNA appeared in the nucleus and membrane of oocytes and mature ova in the experimental group.

**Figure 6:** *In situ* hybridization of *Hctra2* gene in testes and ovaries in *H. cumingii*. **(A)** testes stained with HE. **(B)** Male control group. The sense probes acting on testes. **(C)** Male experience group. The antisense probes acting on testes. **(D)** Ovaries stained with HE. **(E)** Female control group. The sense probes acting on ovaries. **(F)** Female experience group. The antisense probes acting on ovaries. Fc, follicles; Sg, spermatogonia; Sc, spermatocyte; St, spermatid; Sp, sperm; Og, oogonium; Oc, oocyte; and Mo, mature ovum.

### The Expression Profile of *Hctra-2*, *Hcfem-1b*, and *Hcdmrt* After RNAi

We studied the role of *Hctra-2* in the sex regulation of *H. cumingii* by RNAi. The dsRNA transcribed and synthesized *in vitro* was injected into the gonads of *H. cumingii*. The results showed that the silencing efficiency of the dsHctra-2 was 70.6% in males and 55.8% in females (Figures 7A,B), which indicated that the dsRNA-mediated gene silencing was effective. We also observed the changes in expression of *Hcfem-1b* and *Hcdmrt* after *Hctra-2* knockout. Compared with the negative control group, the expression level of the *Hcfem-1b* in testes and ovaries decreased significantly, and the silencing efficiency reached 79.9% in males and 79.0% in females (Figure 7C,D). The expression level of the *Hcdmrt* in the male gonads of the experimental group was 44.7% lower than that of the control group (Figure 7E), and the expression level in female gonads was 16.7% higher than that in the control group (Figure 7F).

**Figure 7:** Effects of dsHctra-2 injection on the expression of *Hctra-2*, *Hcfem-1b*, and *Hcdmrt* genes in testes and ovaries of *H. cumingii*. dsGFP, treated with dsGFP and used as RNAi control group; dsHctra-2, treated with dsRNA of *Hctra-2* as RNAi experiment group. **(A)** The expression of *Hctra-2* gene in testes. **(B)** The expression of *Hctra-2* gene in ovaries. **(C)** The expression of *Hcfem-1b* gene in testes. **(D)** The expression of *Hcfem-1b* gene in ovaries. **(E)** The expression of *Hcdmrt* gene in testes. **(F)** The expression of *Hcdmrt* gene in ovaries. Results are expressed as mean ± SD, and significance of comparison is defined as *p* < 0.05 (^*^) or *p* < 0.01 (^**^) by Student’s *t*-tests.

## Discussion

In this study, we cloned and identified 1867 bp of the *Hctra-2*, including 881 bp 3'-UTR, 92 bp 5'-UTR and 894 bp ORF corresponding to 297 amino acids. *Hctra-2* has a conserved RRM domain (98 amino acids) and linker region (17 amino acids), but only one RS domain (RS1) contains 61 amino acids (Figure 1). The RNP-1 and RRM domains are generally considered to be involved in the recognition of single-stranded RNA and can affect many pre-mRNA selective splicing (Kim et al., 2000; Lee et al., 2017). Like in the Anastrepha fruit flies, the RRM domain of TRA-2 protein confers the *tra-tra2* complex to interact with *tra* and *dsx* pre-mRNAs to regulate sex-specific splicing (Martín et al., 2011). RS domain is rich in serine and arginine dipeptides (Zhang and Sun, 2008), its main function is to mediate splice site recognition and splicing regulation, and its potency is proportional to the number of repeats of RS dipeptides (Philipps et al., 2003; Long and Caceres, 2009). This indicates that the RS and RRM domains in *Hctra-2* endow it with a certain splicing function. The linker region is a characteristic domain of TRA-2 proteins (Dauwalder et al., 1996). We compared the putative HCTRA-2 protein of *H. cumingii* with *M. coruscus*, *C. gigas*, *M. yessoensis*, and *P. maximus.* Figure 2 shows the alignment of these TRA2 proteins with different numbers of amino acids: *H. cumingii* 297, *M. coruscus* 289, *C. gigas* 298, *M. yessoensis* 324, and *P. maximus* 232. This difference in the number of amino acids was caused by changes in the sequence of TRA-2 amino acids except for the RRM domain and the linker (78 and 17 amino acids, respectively). The homology and conservation of the RRM domain and linker domain in these species suggest the functional similarity of the *tra-2* in bivalves. Compared with other species, the linker sequence of HCTRA-2 amino acid has no RS2 domain behind it, which is similar to the *Estra-2c* of *Eriocheir sinensis* (Luo et al., 2017). The absence of the RS2 domain in *Hctra-2* indicates a weak ability to recognize in the precursor mRNAs.

The expression pattern of *Hctra-2* in different tissues and development stages was analyzed by qRT-PCR. Firstly, the tissue distribution showed that the *Hctra-2* expression in gonads was higher than in somatic tissues. And *Hctra-2* showed sexual dimorphism in gonads (Figure 4). The *Hctra-2* expression level in the testis was significantly higher than that in the ovary. This expression pattern is consistent with that of *M. nipponense* in Arthropoda (Wang et al., 2019). It suggests that *Hctra-2* may play a potential regulatory role in gonadal development of *H. cumingii*. But in many other species, *tra-2* has a high expression pattern of ovary, such as *P. chinensis* (Li et al., 2012), *Aedes albopictus* (Li et al., 2019), *E. chinensis* (Luo et al., 2017), and aquatic firefly (*Sclerotia aquatilis*; Nguantad et al., 2020). The different expression patterns of *tra-2* indicate that its regulation of gonadal development is different among species.

The transcripts changes of the *Hctra-2* were further observed during embryonic development and early gonadal development (Figure 5). During embryonic development, the expression of *Hctra-2* was high at fertilized eggs, peaked at day 3, and then decreased. Studies based on the embryonic development of *H. cumingii* showed that the embryo on the third day after fertilization is in cleavage stage (Hong et al., 2007). Interestingly, *Mntra-2a* was also highly expressed in the cleavage stage of *M. nipponense* embryos (Wang et al., 2019). This indicates that *Hctra-2* is very active in embryo division. In a study of *Bactrocera dorsalis*, the expression level of *tra* was increased at the fifteenth hour of embryonic development, suggesting that sexual identity may be established at this stage of embryogenesis (Hong et al., 2007). We speculate that *Hctra-2* may be involved in sex determination at early embryonic stage. In the early stage of gonadal development, *Hctra-2* showed a slight increase at 4 months of age (Figure 5). Ting (2016) found that the gonad tissue of *H. cumingii* began to appear around 5 months of age, suggesting that *Hctra-2* may be involved in the regulation of early gonad development.

The histological location of *Hctra-2* in gonad was analyzed by ISH. *Hctra-2* mRNA was detected in spermatogonia and spermatocytes in the testes (Figure 6C) and in the membrane and nucleus of ovary oocytes and mature ova (Figure 6F). The expression position of *Hctra-2* signals is similar to that of *tra-2* in *M. nipponense* (Wang et al., 2019). These results showed that *Hctra-2* was closely related to spermatogonia proliferation, meiosis of spermatocytes and oocytes, and ova maturation, further confirming that *Hctra-2* was involved in the gonadal development of *H. cumingii*. In addition, no *Hctra-2* mRNA signal was observed in sperm, while in egg, the signals were concentrated in the nucleus and cell membrane. This suggests that the high expression of *Hctra-2* in the fertilized egg is caused by the ova. In *Nasonia vitripennis*, *Nvtra2* was also found in early embryos (<3 h old), suggesting that the mother provides *Nvtra2* to the egg and is critical for embryo viability (Geuverink et al., 2017). Studies of *Bdtra-2* of *Bactrocera dorsalis* have shown that *Bdtra-2* transcripts are contributed maternally and activated by the zygote in the developing embryos (Laohakieat et al., 2020). Therefore, we hypothesized that in *H. cumingii*, *Hctra-2* might be provided by the mother and involved in embryo sex determination during cleavage. However, whether *Hctra-2* is a key gene involved in sex determination needs to be further verified.

In this study, *Hctra-2* was silenced by RNAi to explore further the role of *Hctra-2* in the sex regulation of *H. cumingii*. After injection of *Hctra-2* dsRNA, the expression of *Hcfem-1b* and *Hcdmrt* was observed (Figure 7). These two genes were selected because we know that *tra* is upstream of *fem* in *C. elegans* sex determination process. The activity of TRA-2 protein can directly determine whether it interacts with the FEM protein complex, thus influencing the sex of *C. elegans* (Zanetti and Puoti, 2013). Secondly, in most insects, *tra* forms a conserved central axis of sex determination (Verhulst et al., 2010) and plays a key role in sex determination and maintenance by regulating *dsx* mRNAs (Shukla and Palli, 2013). Both *doublesex and mab-3-related transcription factor* (*dmrt*) and *dsx* belong to the *dmrt* family, and their roles in sex determination and differentiation have been widely studied (Mawaribuchi et al., 2019; Panara et al., 2019). In addition, our previous study identified the homologous genes of *Hcfem-1b* (Wang et al., 2021) and *Hcdmrt* (Ge et al., 2020) of *fem* and *dmrt*. Therefore, we wonder whether there is such upstream or downstream regulatory relationship in *H. cumingii*? With this conjecture in mind, we used RNAi to investigate the interaction of *tra-2*, *fem* and *dmrt* in the regulation mechanism in *H. cumingii*.

RNA interference of *Hctra-2* in both female and male mussels caused the down-regulation of *Hcfem-1b* expression (Figures 7C,D). This indicates that *Hcfem-1b* was downstream of *Hctra-2* and maintained the consistency of synergistic changes with it. However, when the expression of *Hcdmrt* was detected, it was found that the *Hcdmrt* was significantly decreased in males (Figure 7E) and increased in females (Figure 7F). In *Bemisia tabaci*, RNAi with *Bttra2* also affects the expression of *Btdsx*. And, the silencing of *Bttra2* or *Btdsx* resulted in male genital deformities (Guo et al., 2018). We were also found that *Cqdsx* was significantly reduced in the RNAi of *CqTra2* in redclaw crayfish (Cai et al., 2020). These results indicate that *Hcdmrt* is also regulated by *Hctra-2*, but the regulation is different between the sexes. So, is there a regulatory relationship between *Hcfem-1b* and *Hcdmrt*? Here, we propose a hypothesis, and its correctness needs further explored. We found that *dsx* is regulated by *fem* in honeybee sex determination process. Honeybee sex is determined by the heterozygosity of complementary sex determiner (*csd*; Beye et al., 2003; Gempe and Beye, 2011). The *csd* of honeybee is homologous with the drosophila *tra* (Liu et al., 2012). In females, *csd* can produce active CSD protein, which can cleave *fem* to produce functional FEM protein and then promote female splicing of *dsx* transcript and induce female development. On the contrary, the males lack active CSD protein, the *fem* transcripts are spliced into male form, *dsx* pre-mRNA is spliced into the male expressing DSX protein, and the individual develops toward male (Beye et al., 2003; Beye, 2004). Moreover, combined with the silencing efficiency of the genes, the silencing efficiency of *Hcfem-1b* in testes and ovaries was 79.9 and 79.0%, respectively (Figures 7C,D). The silencing efficiency of *Hcdmrt* in testes was 44.7% (Figure 7E) and increased by 16.7% in ovaries (Figure 7F). Thus, *Hcfem-1b* has a higher silencing efficiency, and it is most likely to be directly downstream of *Hctra-2*, while *Hcdmrt* is indirectly downstream of it. Therefore, we boldly speculate that there is a cascading regulatory relationship among these three genes, namely, *Hctra-2* > *Hcfem-1b* > *Hcdmrt*. The difference in this regulatory relationship between males and females is the effect of *Hcfem-1b* on *Hcdmrt*. *Hcfem-1b* may positively regulate *Hcdmrt* in males and negatively regulate *Hcdmrt* in females. But at present, this is our preliminary guess, and the specific way of regulation and its role in gender regulation is our goal in the next stage.

## Conclusion

In this study, the full length of *Hctra-2* of *H. cumingii* was cloned. The results of gene sequence analysis and multiple sequence alignment showed that *Hctra-2* was highly conserved in RRM domain and linker region, and the amino acid sequence similarity among different species was high. The phylogenetic tree showed that *tra-2* was closely related to mollusks. The qRT-PCR results indicated that *Hctra-2* may play an important role in gonadal development and early embryonic development. The probe signal of *Hctra-2* mRNA was found in both male and female gonads, which further indicated that *Hctra-2* was involved in gonadal development. RNAi experiments explored the relationship between two sex-related genes (*Hcfem-1b* and *Hcdmrt*) and *Hctra-2*. We speculated that there was a cascade regulatory relationship between them, and the way of action was different between males and females. However, the specific way of this regulatory relationship and its impact on gender regulation still to be further studied.

## Data Availability Statement

The datasets presented in this study can be found in online repositories. The names of the repository/repositories and accession number(s) can be found at: https://www.ncbi.nlm.nih.gov/genbank/, MH931228.

## Ethics Statement

The animal study was reviewed and approved by the Institutional Animal Care and Use Committee (IACUC) of Shanghai Ocean University, Shanghai, China.

## Author Contributions

XW completed the sample collection. YW and JG conceived and designed the experiments, analyzed the data, interpreted the results, and wrote the manuscript. GW and JL provided feedback on discussion and results. All authors have given approval to the final version of the manuscript.

### Conflict of Interest

The authors declare that the research was conducted in the absence of any commercial or financial relationships that could be construed as a potential conflict of interest.

## Footnotes

^1^https://www.ncbi.nlm.nih.gov/orffinder/

^2^https://blast.ncbi.nlm.nih.gov/Blast.cgi

^3^http://www.cbs.dtu.dk/services/TMHMM/

^4^http://www.cbs.dtu.dk/services/SignalP/

^5^https://web.expasy.org/protparam/

## Abbreviations

*tra-1 and tra-2*: *transformer-1 and transformer-2*
qRT-PCR: quantitative real-time reverse transcription PCR
RNAi: RNA interference
*fem-1*, *fem-2*, and *fem-3*: *feminization-1, feminization-2, and feminization-3*
*dmrt*: *doublesex and mab-3-related transcription factor*
*foxl2*: *forkhead box l2*
*her-1*: *hermaphroditization-1*
*cul-2*: *cullin 2*
*dsx*: *doublesex*
*fru*: *fruitless*
*sxl*: *sex lethal*
dsRNA: double-stranded RNA
ssRNA: single-stranded RNA
ORF: open reading frame
UTR: untranslated region
HE: hematoxylin-eosin
RRM: RNA recognition motif
csd: complementary sex determiner
Fc: follicles
Sg: spermatogonia
Sc: spermatocyte
St: spermatid
Sp: sperm
Og: oogonium
Oc: oocyte
Mo: mature ovum
ISH: *in situ* hybridization
